The article "Investigation of changes in the activity and function of dry eye-associated brain regions using the amplitude of low-frequency fluctuations method" was published in 2022. Journal: Biosci Rep.

# Investigation of changes in the activity and function of dry eye-associated brain regions using the amplitude of low-frequency fluctuations method

**DOI:** 10.1042/BSR20210941

**Published:** 2022-01-11

**Authors:** Tie Sun, Hui-Ye Shu, Jie-Li Wu, Ting Su, Yu-Ji Liu, Li-Juan Zhang, Qiu-Yu Li, Yi-Cong Pan, Qian-Min Ge, Yi Shao

**Affiliations:** 1 Department of Ophthalmology, The First Affiliated Hospital of Nanchang University, Jiangxi Center of National Ocular Disease Clinical Research Center, Nanchang 330006, Jiangxi, People’s Republic of China; 2 Eye Institute of Xiamen University, Fujian Provincial Key Laboratory of Ophthalmology and Visual Science, Medical College of Xiamen University, Xiamen 361102, Fujian Province, People’s Republic of China; 3 Department of Ophthalmology, Massachusetts Eye and Ear, Harvard Medical School, Boston 02114, MA, U.S.A.; 4 Department of Ophthalmology, Guangfeng People’s Hospital, Shangrao 334000, Jiangxi, People’s Republic of China

**Keywords:** amplitude of low frequency fluctuations, dry eye, spontaneous brain activity

## Abstract

**Objective:** The local characteristics of spontaneous brain activity in patients with dry eye (DE) and its relationship with clinical characteristics were evaluated using the amplitude of low-frequency fluctuations (ALFF) method.

**Methods:** A total of 27 patients with DE (10 males and 17 females) and 28 healthy controls (HCs) (10 males and 18 females) were recruited, matched according to sex, age, weight and height, classified into the DE and HC groups, and examined using functional magnetic resonance imaging (fMRI) scans. Spontaneous brain activity changes were recorded using ALFF technology. Data were recorded and plotted on the receiver operating characteristic (ROC) curve, reflecting changes in activity in different brain areas. Finally, Pearson correlation analysis was used to calculate the potential relationship between spontaneous brain activity abnormalities in multiple brain regions and clinical features in patients with DE. GraphPad Prism 8 (GraphPad Software, Inc.) was used to analyze the linear correlation between the Hospital Anxiety and Depression Scale and ALFF value.

**Results:** Compared with HCs, the ALFF values of patients with DE were decreased in the right middle frontal gyrus (MFG)/right inferior orbitofrontal cortex (OFC), left triangle inferior frontal gyrus, left MFG, and right superior frontal gyrus. In contrast, the ALFF value of patients with DE was increased in the left calcarine.

**Conclusion:** There are significant fluctuations in the ALFF value of specific brain regions in patients with DE versus HCs. This corroborates previous evidence showing that the symptoms of ocular surface damage in patients with DE are related to dysfunction in specific brain areas.

## Introduction

Dry eye (DE) is a common disease and is defined as a multifactorial disease of tears and ocular surface, leading to a series of symptoms such as visual disturbance, discomfort, and tear film instability. This condition may damage the ocular surface and is often accompanied by increased tear film osmotic pressure and subacute ocular surface inflammation [1]. Its incidence ranges from 5 to 34% worldwide [2]. According to existing research estimates, approximately 6.8% of the American adult population has been diagnosed with DE. However, it is estimated that another 2.5% of adult Americans may be undiagnosed despite experiencing DE symptoms [3]. The prevalence of DE also increases significantly with age. The pathogenesis of DE includes tear film hypertonicity, ocular surface inflammation, and lacrimal gland inflammation. Clinically, DE can be divided into two subtypes: reduced tear secretion (DE with insufficient water content) and increased tear evaporation (DE with excessive evaporation).

The systematic diagnosis and monitoring of DE should include detailed medical history recording, comprehensive spectroscopic examination, and additional examinations. Commonly used subjective scales include the Ocular Surface Disease Index and the Symptom Assessment in Dry Eye. The former is a questionnaire used to assess symptom development in the previous week. The score ranges between 0 and 100 (higher scores indicate more serious disease). The latter assesses the severity and frequency of DE (rated by patients) using a visual analog scale [4]. These tools can be used in conjunction with clinical examination results. However, thus far, few randomized controlled treatment trials for DE have been performed.

The basic principles of magnetic resonance have been investigated for >70 years and have been the backbone of medical imaging for >40 years [5]. Currently, magnetic resonance imaging (MRI) is a useful non-invasive technique in diagnostic medicine and biomedical research, particularly for evaluating the structure, function, and neurochemical properties of the brain.

Functional magnetic resonance imaging (fMRI) is an emerging neuroimaging method. Its principle is to use MRI to measure changes in hemodynamics caused by neuronal activity. At present, it is mainly used to study the brain or spinal cord of humans and animals [6]. Neurons do not store the glucose and oxygen required for energy; thus, the energy utilized for nerve activation must be rapidly replenished. Through the process of hemodynamic reaction, the blood supplies more oxygen than the nerves need. Due to the difference in permeability between oxygenated and deoxygenated hemoglobin, the changes in the volume of oxygenated and hypoxic blood cause disturbances in the magnetic field which can be detected by MRI. Through repetition of certain thoughts, actions, or experiences, statistical methods can be used to determine the brain areas in which signal changes occur during the process. Using this approach, it is possible to identify the brain areas involved in performing these thoughts, actions, or experiences (e.g., the visual pathway from the retina to the cortex and the spatial organization of the brain). These analyses can help clarify the pathogenesis of eye diseases [7]. The concept of blood oxygen level-dependent imaging was first proposed by Ogawa et al. in 1990 [8]. Most fMRI studies use the blood oxygen-level dependent imaging method to detect response areas in the brain. Amplitude of low-frequency fluctuations (ALFF) is an indicator of local spontaneous neuronal activity when the blood oxygen level depends on the signal at low frequencies. It is regarded as a highly accurate and sensitive measurement method [9]. The etiology of DE is multifactorial, often associated with depression, anxiety, stress etc., as well as neurological and mental diseases [10]. The use of drugs for the treatment of mental illness can also have an impact on DE. Therefore, DE may be related to the nervous system and brain function. Previous studies have successfully used the ALFF method to assess brain activity in retinal vein occlusion [11], optic neuritis [12], acute eye pain [13,33], Alzheimer’s disease [31], amblyopia [32], depression [34], and diabetic retinopathy [35] (Table 4).

The present study used the ALFF method to evaluate the intrinsic brain activity of patients with DE and healthy controls (HCs), and the correlation between intrinsic brain activity and clinical manifestations. In this investigation, it was assumed that patients with DE may have abnormal activities in some brain regions.

## Materials and methods

### Subjects

A total of 27 patients with DE who met the inclusion criteria stated below were recruited at the Department of Ophthalmology, The First Affiliated Hospital of Nanchang University (Nanchang, China) between March 2018 and June 2020. During this period, 28 HCs matched to those included in the DE group in terms of sex, age, and education level were recruited to form the control group. The research was conducted in accordance with the Declaration of Helsinki and approved by the Ethics Committee of The First Affiliated Hospital of Nanchang University. All participants understood the purpose, content, and risks of the study, and provided written informed consent.

### Inclusion and exclusion criteria

The diagnostic criteria for DE were symptoms such as DE, foreign body sensation, burning sensation, cracking, itching, photophobia, blurred vision, and asthenopia, with: (1) rupture time < 10 s; (2) Schirmer I < 10 mm/5 min; and (3) positivity for fluorescein staining (Figure 1).

**Figure 1:** Typical fundus photographs of dry eye disease

The selection criteria for the subjects were: (1) meeting the diagnostic criteria for lacrimal DE; (2) age: 20–75 years; (3) no treatment with other medication or withdrawal period for >2 weeks; and (4) informed consent to receive treatment.

The exclusion criteria for patients with DE were: (1) conjunctival scar, atresia of the lacrimal gland, or complete atrophy of the accessory lacrimal gland; (2) other obvious conjunctival, corneal, and iris disease; (3) pregnancy or lactation; and (4) history of drug abuse.

All HCs met the following criteria: (1) no brain parenchymal abnormalities found on MRI; (2) no eye disease, no visual impairment, and uncorrected vision (visual acuity > 1.0); (3) normal mental health and no abnormalities in neurological examination; and (4) no contraindications to MRI.

### MRI parameters

All subjects were scanned with a 3-Tesla magnetic resonance scanner (Trio, Siemens, Munich, Germany). They were instructed to keep their eyes close d, but to remain awake and relaxed until the end of the scan. The relevant data were obtained using a three-dimensional spoiled gradient-recalled echo sequence in the MRI. The imaging parameters of the T1 and T2 sequences for 176 traverse images were as follows: repetition time (TR) = 1900 ms; echo time (TE) = 2.26 ms; thickness = 1.0 mm; gap = 0.5 mm; acquisition matrix = 256 × 56; field of view = 250 × 250 mm; and flip angle = 9°. The imaging parameters for 240 functional images were as follows: TR = 2000 ms; TE = 30 ms; thickness = 4.0 mm; gap = 1.2 mm; acquisition matrix = 64 × 64; flip angle = 90°; field of view = 220 × 220 mm; and 29 axials. The scanning times were 5 and 10 min, respectively.

### fMRI data processing

We used the MRIcro software (https://www.mccauslandcenter.sc.edu/crnl/mricro) to identify valuable data to be collected. To maintain magnetization equilibrium, we also discarded the first ten time points. We employed the Data Processing Assistant for Resting-State fMRI (DPARSF) software to analyze the Digital Imaging Communications in Medicine (DICOM) images, performed correction for head movement, normalized the spatial position and slice time, and performed full-width smoothing with a Gaussian kernel of 6 × 6 × 6 mm^3^ at half-maximum based on the resting state-fMRI data analysis toolkit (REST) software and Statistical Parametric Mapping software (SPM; The MathWorks, Inc.) Subjects with ≥1.5-mm exceeding shift in x, y, or z or 1.5 angular motion were eliminated. After that, the head motion artifacts were corrected, and the interference effect was eliminated using linear regression. Following correction for head movement, a standard echo plane image template was used to ensure that the collected data reached the standards of the Montreal Neurological Institute (Montreal, Canada). The data were further processed using a Gaussian kernel to calculate the ALFF. Additionally, the fMRI images were detrended and bandpass-filtered (0.01–0.08 Hz) to increase the accuracy of images and reduce the deviation caused by breathing or cardiac noise.

### Statistical analysis

Independent sample *t* tests and chi-squared tests were performed using the Statistical Package for the Social Sciences software (SPSS version 23.0; IBM Corporation, Armonk, NY, U.S.A.) to determine differences in clinical characteristics. The difference between the average ALFF values of patients with DE and HCs was determined using an independent *t* test and receiver operating characteristic (ROC) curve. In all statistical analyses, a *P*-value <0.05 denoted statistically significant difference.

### Brain-behavior correlation analysis

Specific clusters are calculated from the ALFF values, the REST software divides the brain into different regions of interest (ROIs) based on the voxel value ratio. The average ALFF value for each ROI is the average regional homogeneity of all voxels for that region. The correlation between ALFF values in ROIs and clinical features in patients with ophthalmectomy was evaluated through Pearson’s correlation analysis.

## Results

### Demographics and visual measurements

As shown in Table 1, there were no significant differences in age (*P*=0.839), height (*P*=0.668), weight (*P*=0.724), and body mass index (*P*=0.912) between the two groups.

**Table 1:** Clinical characteristics of patients between dry eye disease and HC groups

Characteristics	DE	HCs	*t* value	*P*-values
Male/female	10/17	10/18	NA	NA
Age (years)	56.13 ± 9.72	55.23 ± 9.18	−0.238	0.839
Weight (kg)	57.24 ± 7.36	58.24 ± 6.97	−0.412	0.724
Height (cm)	165.53 ± 9.28	164.32 ± 6.16	−0.418	0.668
BMI (kg/m^2^)	22.61 ± 1.54	21.93 ± 1.46	−0.049	0.912
Duration of DED (mons)	9.67 ± 3.14	NA	NA	NA
Duration from onset of DED to rs-fMRI scan (mons)	9.42 ± 2.98	NA	NA	NA
Best-correted VA, right	0.95 ± 0.35*	1.15 ± 0.15	−0.512	0.538
Best-correted VA, left	0.85 ± 0.40*	1.05 ± 0.20	−0.648	0.659

Independent *t* tests comparing the two groups (*P<0.05) represented statistically significant differences. Abbreviations: BMI, body mass index; DED, dry eye disease; NA, not applicable; rs-fMRI, resting-state functional magnetic resonance; VA, visual acuity.

### ALFF differences

Compared with the HC group, the ALFF values of the right middle frontal gyrus (MFG)/right inferior orbitofrontal cortex (OFC), left triangle inferior frontal gyrus (IFG_Tri), left MFG, and right superior frontal gyrus were significantly reduced in the DE group (*P*<0.05), whereas that of the left calcarine was significantly increased (*P*<0.05) (Figures 2 and 3, Table 2).

**Figure 2:** Spontaneous cerebral activity in dry eye disease patients and HC There were significant differences in brain activities of Frontal_Mid_R/Frontal_Inf_Orb_R, Frontal_Inf_Tri_L, Frontal_Mid_L, Frontal_Sup_R, and Calcarine_L. The red or yellow denotes increased ALFF values, and the blue areas indicate decreased ALFF values, respectively (P,0.01 for multiple comparisons using Gaussian random field theory (z.2.3, P,0.01, cluster. 40 voxels, Alphasim corrected)).

**Figure 3:** Mean ALFF values between the dry eye disease and HC groups in the different regions of the brain

**Table 2:** Brain areas with significantly different ALFF values between dry eye disease and HCs groups

Brain areas	MNI coordinates			Number of voxels	*t* value
	x	y	z		
HCs > DED					
Frontal_Inf_Orb_R (aal)	39	39	9	249	5.8613
Frontal_Inf_Tri_L (aal)	−39	27	21	95	4.7743
Frontal_Mid_L (aal)	−33	36	39	44	4.4244
Frontal_Sup_R (aal)	27	45	45	45	4.7222
HCs < DED					
Calcarine_L (aal)	−6	75	9	44	−3.9692

### Correlation analyses

In the DE group, the mean hospital anxiety and depression scale-depression (HADS) score was negatively correlated with the ALFF signal values of the Frontal_Mid_R /Frontal_Inf_Orb_R (r = −0.5094, *P*=0.056; Figure 5A), the mean HADS score was negatively correlated with the ALFF signal values of the Frontal_Sup_R (r = −0.8747, *P*<0.0001; Figure 5B). The LogMAR score in the DE group was negatively correlated with the ALFF signal values of the Frontal_Mid_L (r = −0.3830, *P*=0.0443; Figure 5C). The LogMAR score in the DE group was negatively correlated with the ALFF signal values of the Frontal_Mid_L (r = −0.3830, *P*=0.0443; Figure 5D).

### ROC curves

ROC curves were used to evaluate the average ALFF value of the right MFG/right inferior OFC, left IFG_Tri, left MFG, right superior frontal gyrus, and left calcarine. The areas under the curves for the ALFF values were as follows: right MFG/right inferior OFC (0.909), left IFG_Tri (0.925), left MFG (0.878), right superior frontal gyrus (0.825) (Figure 4A), and left calcarine (0.788) (Figure 4B).

**Figure 4:** ROC curve analysis of the mean ALFF values for changed areas The AUCs of ALFF values were as follows: Frontal_Mid_R/Frontal_Inf_Orb_R (0.909), Frontal_Inf_Tri_L (0.925), Frontal_Mid_L (0.878), Frontal_Sup_R (0.825), (**A**), Calcarine_L (0.788) (**B**). Abbreviation: AUC, area under the curve.

**Figure 5:** Correlations between the mean ALFF value and HADs/LogMAR (**A**) The HADS score in the DE group was negatively correlated with the ALFF signal values of the Frontal_Mid_R/Frontal_Inf_Orb_R (r = −0.5094, *P*=0.056). (**B**) The HADS score in the DE group was negatively correlated with the ALFF signal values of the Frontal_Sup_R (r = −0.8747, *P*<0.0001). (**C**) The LogMAR score in the DE group was negatively correlated with the ALFF signal values of the Frontal_Mid_L (r = −0.3830, *P*=0.0443). (**D**) The LogMAR score in the DE group was negatively correlated with the ALFF signal values of the Frontal_Mid_L (r = −0.3830, *P*=0.0443). Abbreviation: LogMAR, logarithm of the minimum angle of resolution.

## Discussion

To our knowledge, this is the first study to determine whether there are differences in ALFF values in brain regions of patients with DE versus HCs. Moreover, the study sought to determine the location of these regions and the mechanisms involved in these changes in ALFF values.

### Analysis of low ALFF values in the DE group

The areas that showed lower ALFF values were the right OFC/left MFG, left IFG_Tri, right MFG, and right dorsolateral superior frontal gyrus (Figure 6).

**Figure 6:** Significant differences in spontaneous brain activity between the dry eye disease and HC groups

Brodmann first described the anatomical features of the OFC area in 1909. Since then, animal disease model studies and imaging have shown that the prefrontal cortex (PFC) plays an important role in assessing patient prognosis and surgical risk. At present, the understanding of the prefrontal lobe has gradually penetrated into the field of behavior and cognitive function. For determining ROIs from a functional point of view, the right OFC refers to the area of the frontal cortex that participates in rewards and decision-making. The determination of ROIs from the perspective of surgical operation is based on the anatomical structure. The OFC refers to the cortex of the frontmost cerebral cortex, the posterolateral IFG, the posterior insula, and the medial straight back [14]. Neurofunctional research data have shown that the OFC and its white matter fiber network are involved in human executive functions [15]. They can also participate in the regulation of emotional separation [16] and depressive tendency [17] of individuals. Information on object vision passes through the temporal lobe cortex visual area and is input into the OFC. The OFC visual neurons respond differently to different objects or images, and the results are linked to reward-related functions [14].

The findings of the present study indicate that visual fatigue, visual foreign body sensation, dryness, and other visual impairment symptoms of patients with DE are, to a certain extent, related to the OFC. We conjecture that a decrease in the ALFF value of patients with DE may indicate that the OFC is damaged, the mental and emotional states of these individuals are poor, and their inhibitory control ability is weakened. Moreover, we should pay attention to the link between the underlying mechanism of depression and the low activity of the right OFC. In the present study, the HADS score in the DE group was negatively correlated with the ALFF signal values of the OFC. DE is a recognized risk factor for anxiety and depression. DE patients were more prone to anxiety than the general population, and in a study of 89 DE patients, tested using ‘Zung Anxiety Self-Assessment Scale (SAS)’, ‘Zung Depression Self-Assessment Scale (SDS)’, and ‘Eye Table Disease Index (OSDI)’, found that DE patients were more prone to anxiety and depression [36], Therefore, we suppose that the DE may damage the OFC by causing depression, which may be a possible reason for ALFF change. In such cases, attention should be paid to strengthening psychological counseling and nursing.

The MFG is located between the superior frontal sulcus and the subfrontal sulcus, and is connected to the anterior orbital gyrus on the lower surface of the hemisphere. It is closely related to language [18], working memory [19], and other functions. The visual and selective attention tasks will also induce changes in MFG-related network nodes [20]. In a study of patients with primary angle-closure glaucoma, Huang et al. found that both sides of the MFG had lower HCs in the ALFF area [21]. The average ALFF signal of the MFG was negatively correlated with the average thickness of the contralateral retinal nerve fiber layer [21]. In addition, a previous study showed that patients with early blindness may show reduced functional connectivity between the right temporal plane and the frontal lobe [22]. This may affect or even hinder the transmission of visual signals. Similarly, DE may lead to decreased frontal lobe activation. The present study found that the ALFF value of MFG in patients with DE was significantly reduced, suggesting an association between the MFG and the clinical symptoms of patients with DE.

The IFG_Tri is a part of the IFG located between the ascending branch and the anterior branch of the lateral groove. It is the central area of Broca’s sports language area and participates in the evaluation of sensory and emotional information [23]. Research has shown that there is a certain connection between this area and Parkinson’s syndrome [24]. Yu et al. reported that the ALFF value of the left IFG was significantly reduced in patients with diabetic retinopathy [25]. This is consistent with the present findings. We hypothesized that a decrease in the ALFF value of the left IFG_Tri may indicate abnormal brain activity in this brain area. Therefore, it can be speculated that DE may cause a series of language barriers and social and psychological problems in patients.

The PFC refers to the entire frontal cortex except for the primary and secondary motor cortices. The dorsolateral PFC is a subarea of the PFC, which is related to cognition, emotion, pain, and behavior management [26]. In particular, it participates in the executive control of saccades [27]. A decrease in the ALFF value of the dorsolateral PFC may indicate that the burning sensation, eye pain, and soreness of the eyes of patients with DE are serious, which is the result of compensation.

### Analysis of higher ALFF values in the DE group

Calcarine fissure is an approximately horizontal arcuate deep groove on the inner surface of the occipital lobe, which is located at the back of the inner side of the hemisphere [28]. Nayomi et al. reported that visual defects and reduced multifocal standard visual evoked potentials (VEPs) related to changes in the bilateral calcarine sulcus. Nobusada et al. demonstrated that the relationship between the optic nerve tract or calcarine fissure and occipital lobe tumors may lead to postoperative visual field defects [29].

The visual cortex, which is located around the talc fissure of the occipital lobe, is part of the cerebral cortex that is mainly responsible for the processing of visual information. It is a typical sensory granular cortex (koniocortex) that accepts visual information input from the lateral geniculate body of the thalamus. The human visual cortex includes the primary visual cortex (V1) and extrastriate cortex, such as V2, V3, V4, V5 etc. The V1 is also termed the striated zone, including the cortical area, cuneiform lobe, and lingual gyrus on both sides of the calcarine sulcus. It plays an important role in perceiving and integrating visual information, and is often referred to as the visual contact area [30]. It can be inferred that the visual impairment of patients with DE is largely related to increased ALFF values of the left calcarine sulcus and surrounding cortex. In other words, the symptoms (e.g., blurred vision and fluctuation of vision) in patients with DE directly or indirectly lead to the abnormal activation of the left calcarine sulcus and surrounding cortex. However, it should be noted that the depth and length of the calcarine sulcus change independently in the human brain. Hence, the size of the V1 area cannot be judged based on the length and depth of the calcarine sulcus.

## Limitations

The present study had certain limitations. Firstly, the number of the participants is relatively small. Additional studies involving a larger population are warranted to verify the present findings. Secondly, the fMRI scan time in patients with DE differed; these individual differences may undermine the accuracy of our analysis. Thirdly, our study only demonstrated the existence of the relationship between changes of ALFF values in specific brain regions and DE. However, whether DE causes the activity changes in the brain or patients who have suffered brain dysfunction are inclined to DE is still vague. We therefore expect a series of molecular experiments to elucidate further mechanisms. Despite these limitations, the present study provides information on changes in activity in different areas of the brain.

## Conclusion

In summary, our research data show that patients with DE have abnormal activities in the right MFG/right inferior OFC, left IFG_Tri, left MFG, right superior frontal gyrus, and left calcarine. The change in ALFF value reflects the activity of the brain area (Table 3). The dysfunction in these brain regions may be related to the pathogenesis of DE. These findings provide a basis for studying the pathogenesis of DE and new ideas for clinical diagnosis and treatment.

**Table 3:** Brain regions with altered ALFF values and the potential impacts

Brain regions	Experimental	Brain function	Anticipated results
Frontal_Inf_Orb_R	DED < HCs	Executive function, reward mechanism, emotional separation, depressive tendency	Hypoactivity of this area
Frontal_Inf_Tri_L	DED < HCs	Language comprehension, evaluation of sensory and emotional information	Language disability
Frontal_Mid_R/ Frontal_Mid_L	DED < HCs	Language function, working memory	Decreased efficiency of visual and selective attention tasks
Frontal_Sup_R	DED < HCs	Cognitive, emotional, pain and behavior management	Burning sensation, eye pain, soreness decreased, and function improved
Calcarine_L	DED > HCs	Visual defects, vision function etc.	Visual function improvement

Abbreviation: DED, dry eye disease.

**Table 4:** The ALFF applied in ophthalmology and other diseases

Author	Year	Disease	Brains areas	
			ALFF increased	ALFF decreased
Liu et al. [31]	2018	Alzheimer’s disease	hippocampus	Bilateral inferior cerebellum lobe, bilateral precuneus, and the Cingulum
Liang et al. [32]	2016	Amblyopia	bilateral calcarine, the left middle occipital gyrus, and the left postcentral gyrus	Bilateral precuneus cortex
Pan et al. [33]	2018	Acute eye pain	Right and left parahippocampal gyri and left caudate	Left and right precentral/postcentral gyrus and left precuneus
Zhong et al. [34]	2019	Depression	Right middle occipital gyrus	Bilateral precuneus, posterior cingulate cortex
Wang et al. [35]	2017	Diabetic retinopathy	Bilateral occipital gyrus, right lingual gyrus, and precuneus	Right posterior/anterior cerebellar lobe and the parahippocampal, fusiform, superior temporal, inferior parietal, and angular gyrus

## Data Availability

The datasets generated during and/or analyzed during the current study are available from the corresponding author on reasonable request.

## Abbreviations

ALFF: amplitude of low-frequency fluctuation
DE: dry eye
fMRI: functional magnetic resonance imaging
HADS: hospital anxiety and depression scale-depression
HC: healthy control
MFG: middle frontal gyrus
MRI: magnetic resonance imaging
OFC: orbitofrontal cortex
PFC: prefrontal cortex
ROC: receiver operating characteristic
ROI: region of interest
TE: echo time
TR: repetition time
